# Dysequilibrium of the PTH-FGF23-vitamin D axis in relapsing remitting multiple sclerosis; a longitudinal study

**DOI:** 10.1186/s10020-018-0028-3

**Published:** 2018-05-30

**Authors:** Mark Simon Stein, Gregory John Ward, Helmut Butzkueven, Trevor John Kilpatrick, Leonard Charles Harrison

**Affiliations:** 1 The Royal Melbourne Hospital, Parkville, Australia; 2 Department of Diabetes and Endocrinology, The Royal Melbourne Hospital, Parkville, VIC 3050 Australia; 3 Walter and Eliza Hall Institute of Medical Research, Parkville, Australia; 4 Sullivan Nicolaides Pathology, Brisbane, Australia; 5 Florey Neuroscience Institutes, Parkville, Australia; 6 University of Melbourne, Parkville, Australia; 7 Monash University, Melbourne, Australia

**Keywords:** Multiple sclerosis, Vitamin D, Parathyroid hormone, Fibroblast growth factor 23

## Abstract

**Background:**

Parathyroid glands of people with relapsing remitting multiple sclerosis (RRMS) fail to respond to low serum 25-hydroxyvitamin D (25OHD) and low serum calcium, which are stimuli for parathyroid hormone (PTH) secretion. This led us to hypothesise: that there is suppression of PTH in RRMS due to higher than normal serum concentrations of fibroblast growth factor 23 (FGF23). We therefore sought evidence for dysregulation of the PTH-FGF23-vitamin D axis in RRMS.

**Methods:**

Longitudinal study (winter to summer) with fasting venepunctures. For RRMS subjects who recruited a healthy control (HC) friend, pairs analyses were performed. For each pair, the within-pair difference of the variable of interest was calculated (RRMS minus HC). Then, the median of the differences from all pairs was compared against a median of zero (Wilcoxon) and the 95% confidence interval of that median difference (CI) was calculated (Sign Test).

**Results:**

RRMS had lower winter PTH than HC, *P* = 0.005, (CI -2.4 to 0.5 pmol/L, *n* = 28 pairs), and lower summer PTH, *P* = 0.04, (CI -1.8 to 0.5, *n* = 21 pairs). Lower PTH associates physiologically with lower intact FGF23 (iFGF23), yet RRMS had higher iFGF23 than HC in winter, *P* = 0.04, (CI -3 to 15 pg/mL, *n* = 28 pairs) and iFGF23 levels comparable to HC in summer, *P* = 0.14, (CI -5 to 13, *n* = 21 pairs). As PTH stimulates and FGF23 reduces, renal 1-alpha hydroxylase enzyme activity, which synthesises serum 1,25-dihyroxyvitamin D (1,25(OH)_2_D) from serum 25OHD, we examined the ratio of serum 1,25(OH)_2_D to serum 25OHD. In winter, this ratio was lower in RRMS versus HC, *P* = 0.013, (CI -1.2 to - 0.3, *n* = 28 pairs).

**Conclusions:**

This study revealed a dysequilibrium of the PTH-FGF23-vitamin D axis in RRMS, with lower plasma PTH, higher plasma iFGF23 and a lower serum 1,25(OH)_2_D to 25OHD ratio in RRMS compared with HC subjects. This dysequilibrium is consistent with the study hypothesis that in RRMS there is suppression of the parathyroid glands by inappropriately high plasma concentrations of iFGF23. Studying the basis of this dysequilibrium may provide insight into the pathogenesis of RRMS.

## Background

Vitamin D is synthesised in skin upon exposure to ultraviolet light and converted in the liver to 25-hydroxyvitamin D (25OHD), the main vitamin D metabolite in serum and the clinical indicator of vitamin D nutrition (Parfitt et al. 1982; Hollis 1996). Serum 25OHD is converted in the kidney tubules and immune cells (macrophages, dendritic cells, and potentially B and T lymphocytes) to a very potent form of vitamin D, 1,25-dihydroxyvitamin D (1,25(OH)_2_D), by 1-alpha hydroxylase (Tanaka and DeLuca 1981; Reichel et al. 1987a; Reichel et al. 1987b; Bacchetta et al. 2013; Shimada et al. 2004; Shimada et al. 2005; Enioutina et al. 2009; Carvalho et al. 2017), which is increased by parathyroid hormone (PTH) and reduced by fibroblast growth factor-23 (FGF23) (Tanaka and DeLuca 1981; Bacchetta et al. 2013; Shimada et al. 2004; Shimada et al. 2005; Gattineni et al. 2011). Serum 1,25(OH)_2_D is degraded by renal 24-hydroxylase, which is reduced by PTH and increased by FGF23 (Tanaka and DeLuca 1981; Shimada et al. 2004; Gattineni et al. 2011). PTH and FGF23 thus regulate serum 1,25(OH)_2_D concentrations through opposite effects on synthetic and degradative hydroxylases.

These regulatory pathways include serum 1,25(OH)_2_D itself, which feeds back both on the enzymes 1-alpha-hydroxylase and 24-hydroxylase (Colston et al. 1977) and on the hormones PTH and FGF23. 1,25(OH)_2_D directly stimulates the synthesis of FGF23 by osteoblasts and osteocytes (Shimada et al. 2004; Nguyen-Yamamoto et al. 2017). It can increase the absorption of dietary calcium and phosphate, and higher serum concentrations of calcium and phosphate may feedback to stimulate FGF23 secretion (Shimada et al. 2005; Nguyen-Yamamoto et al. 2017; Quinn et al. 2013). Serum 1,25(OH)_2_D also feeds back directly on the parathyroid glands to reduce PTH synthesis (Silver et al. 1986) and also indirectly by its action to increase serum concentrations of FGF23, which may then further reduce PTH synthesis and secretion (Ben-Dov et al. 2007; Lavi-Moshayoff et al. 2010). Completing another feedback loop, PTH, the secretion of which is reduced by FGF23, in turn stimulates FGF23 synthesis by osteoblasts and osteocytes (Ben-Dov et al. 2007; Lavi-Moshayoff et al. 2010).

FGF23 circulates as an intact molecule (iFGF23), which is cleaved to release a C-terminal fragment (cFGF23) (Razzaque and Lanske 2007; Blau and Collins 2015). FGF23 binds a variety of FGF receptor subtypes, either directly or in conjunction with the Klotho receptor (Gattineni et al. 2011; Razzaque and Lanske 2007; Blau and Collins 2015; Kurosu et al. 2006). A soluble alpha fragment of the Klotho receptor may also circulate and may serve to stimulate FGF23 synthesis (Smith et al. 2012).

In winter, a decrease in sunlight exposure and vitamin D synthesis is associated with an increase in serum PTH, which maintains the serum calcium concentration. In people with relapsing remitting multiple sclerosis (RRMS), Soilu-Hänninen et al. (Soilu-Hänninen et al. 2008) observed that the winter rise in serum PTH was blunted and was associated with lower serum calcium, compared to healthy controls (HC). It appeared that the parathyroid glands of people with RRMS failed to respond to two stimuli for PTH secretion, namely lower concentrations of vitamin D and serum calcium. This led us to hypothesise that there is suppression of PTH in RRMS due to higher than normal serum concentrations of FGF23. In the present study, we sought evidence for dysregulation of the PTH-FGF23-vitamin D axis in RRMS, in a longitudinal study from winter to summer.

## Methods

### Subjects

People with RRMS (aged ≥18 years) were recruited from hospital clinics and through publicity on the MS Australia Victoria website in July–August 2011. They were asked to bring one or more healthy friends (aged ≥18 years) to serve as healthy controls (HC).

The study was approved by the Human Research Ethics Committees of Melbourne Health and Eastern Health, Victoria. All subjects provided written informed consent.

Exclusions to filter out conditions affecting mineral metabolism were:

Pregnancy, breast-feeding, fracture, bone/joint surgery, treatment with raloxifene, alendronate, risedronate, zoledronate, strontium ranelate or teriparetide in the previous 6 months.

Except for the oral contraceptive, treatment with estrogen or progesterone, testosterone, phenytoin, valproate or levetiracetam in the previous 3 months.

Treatment with oral or systemic glucocorticoid in the previous month.

Treatment with furosemide or thiazide diuretic in the previous week.

Inability to ambulate 300 m without assistance of another person.

HC were excluded if a 1st- or 2nd-degree relative had a history of demyelination.

The following were permitted: oral contraceptives, asthma inhalers, over-counter vitamin/mineral supplements.

We sought to enrol at least 20 individuals with RRMS and 20 HC based on the sample size used to report that people with RRMS failed to increase their serum PTH concentrations in winter (Soilu-Hänninen et al. 2008).

Between August 19th-September 28th 2011 subjects had fasting ‘winter’ venepuncture at collection centres of Melbourne Pathology (Sonic Healthcare, Collingwood, Victoria). Venepuncture was performed between 7:30 am–10 am to control for circadian variation in PTH. Subjects were asked to avoid alcohol for at least 24 h before venepuncture. Each RRMS-HC friend pair attended the same centre at the same time and was randomised (via central computer) as to within-pair venepuncture order. They completed questionnaires regarding anthropometrics, personal and family health. Body mass index (BMI) was calculated as weight (kg)/[height (m)]^2^.

Subjects with serum 25OHD < 50 nM were advised that their vitamin D nutrition was suboptimal. They were given their serum 25OHD result to take to their primary care physician with the recommendation that they commence vitamin D3 (1000 IU daily). We did not mandate or monitor such supplementation as we planned to directly measure serum 25OHD on repeat venepuncture.

Subjects were invited to return February 2012 for identical ‘summer’ collections, preserving within-pair venepuncture order.

### Laboratory assays

EDTA blood tubes were centrifuged immediately, as were serum separator tubes after blood had clotted. Plasma for PTH assay was transported at ambient temperature (Glendenning et al. 2002). Remaining plasma and sera were frozen on site then transported for same day general biochemistry analysis or for storage at − 80 C. Melbourne Pathology Central Laboratory (Collingwood, Melbourne) measured serum biochemistry (Modular c701 chemistry analyser; Roche, Mannheim, Germany), plasma human intact PTH (Modular e602 immunoassay analyser; Roche, Mannheim, Germany) with coefficient of variation (CV) = 4.0% (2–50 pmol/L) and serum 25OHD (Liaison analyser in winter, Liaison XL analyser in summer; DiaSorin, Turin, Italy), with CV = 7.5% (40–280 nmol/L). Calcium corrected for albumin (Cacorr) was calculated as total calcium (mmol/L) + (40-albumin [g/L]) × 0.02.

Sullivan Nicolaides Pathology, (Sonic Healthcare, Brisbane, Australia) measured plasma intact FGF23 (iFGF23) by ELISA (CY4000; Kainos Laboratories, Tokyo, Japan) (Yamazaki et al. 2002 and see also Imel et al. 2006 and Smith et al. 2013), with interassay CV = 3% (at mean 71.8 pg/mL) and 4% (at mean 203.3 pg/mL), plasma C-terminal FGF23 peptide (FGF23c) by ELISA (Immunotopics, San Clemente, USA) with interassay CV = 9% (at mean 32.3) and 1% (at mean 293) and plasma soluble alpha klotho (Klotho) by ELISA (IBL, Hamburg Germany), with interassay CV = 4% (at mean 1130.8 pg/mL) and 4% (at mean 1322.3 pg/mL). Serum ferritin was assayed with the Architect kit, (Abbott, Abbott Park, Illinois, USA). Serum 1,25OH_2_D was measured by immunoassay (IDS iSYS, Tyne and Wear, UK).

For ELISAs, summer and winter specimens from each RRMS-HC pair were measured in the same assay (within the same ELISA plate). Laboratory personnel were blind to source of specimens.

## Statistics

The frequencies of characteristics of RRMS and HC subjects were compared by Fisher’s exact test. Cohort median values for biochemical analytes of RRMS and HC subjects were compared by Mann-Whitney test. The 95% confidence intervals (CIs) for differences between cohort medians were calculated by Moods Median Test.

For RRMS subjects who had recruited an HC friend, pairs analyses were performed. For each pair, the within-pair difference of the variable of interest was calculated (RRMS minus HC). Then, the median of the differences from all pairs was compared against a median of zero (Wilcoxon) and the 95% CI of that median difference was calculated (Sign Test).

Modelling (general linear modelling/multiple regression/path analysis) was not performed as bi-directional causality (Ben-Dov et al. 2007) renders such approaches invalid (personal communication, Professor Terry Speed, Bioinformatics Division, Walter and Eliza Hall Institute of Medical Research, Melbourne).

Statistical analyses were performed on Minitab 13.1 and 17 (http://www.minitab.com). Outliers were defined by the Minitab definition, i.e. > 1.5 x interquartile range (IQR) outside the IQR. *P* < 0.05 was considered significant. Hypotheses with an a priori direction, viz. lower PTH, higher FGF23 (RRMS versus HC), were tested one-tailed (Armitage and Berry 1994). Other hypotheses were tested two-tailed.

## Results

55 RRMS and 35 HC subjects were recruited in winter. Their median (IQR) ages were 46.5 (36.5–52.5) and 49.5 (38.5–56.0) years, respectively (*P* = 0.2). RRMS and HC were 71% and 43% female (F), respectively, (*P* = 0.007). Subjects were excluded for non-return of the questionnaire (3 RRMS, 2 HC) and confounding medication (2 HC), leaving 83 winter subjects. Of RRMS, 14 (27%) were on no therapy, 6 (12%) took glatiramer acetate, 26 (50%) interferon-beta, 2 (4%) natalizumab and 4 (8%) fingolimod; 38% were taking vitamin D compared to 16% HC (*P* = 0.02), and 12% were taking calcium compared to 6% HC (*P* = 0.4).

Median (IQR) BMIs were: RRMS 23.9 (21.2–29.2) and HC 26.2 (22.8–29.0) kg/m^2^ (*P* = 0.4). Two RRMS females with outlier BMIs (43.3, 43.0) and 1 RRMS female with BMI 16.9 (not clinically consistent with normal mineral metabolism) were excluded. One female HC had a failed winter venepuncture. This left 79 subjects (49 RRMS, 30 HC) for whom winter plasma PTH and other analytes were studied for cohort analyses. Of these, 61 (38 RRMS, 23 HC) agreed to return for summer venepuncture for measurement of plasma PTH and other analytes. After the above exclusions, 28 RRMS-HC pairs remained for winter analyses and 23 RRMS-HC pairs for summer analyses. We did not ascertain the reasons why some subjects declined to return in summer.

### 25OHD and 1,25(OH)_2_D

Serum 25OHD increased from winter to summer in both RRMS and HC (*P* < 0.01). However, for serum 1,25(OH)_2_D a significant seasonal rise was detected only in the HC (*P* = 0.02) (Fig. 1, Table 1).

**Fig. 1:** Serum 25OHD and serum 1,25(OH)_2_D Individual values (open circles), cohort medians and interquartile ranges (boxes) are plotted for those subjects who had both winter and summer measurement of serum 1,25(OH)_2_D. Serum 25OHD increased from winter to summer in both HC and RRMS subjects. However, only HC demonstrated a significant seasonal rise in serum 1,25(OH)_2_D

**Table 1:** Cohort analyses

Chemical	RRMS median (IQR)	HC median (IQR)	95% CI for difference (RRMS-HC) in medians	*P* value
For 25OHD and PTH, *n* = 49 for RRMS and 30 for HC. For all other analytes below, *n* = 38 for RRMS and *n* = 25 for HC				
Winter 25OHD	58 (40–89)	43 (36–71)	-3 to 32	0.09
Summer 25OHD	87 (70–108)^***^	81 (70–92)^***^	−6 to 18	0.4
Winter PTH	4.5 (3.7–6.0)	5.8 (4.1–6.6)	−1.6 to −0.3	0.02
Summer PTH	4.7 (3.9–5.7)	5.0 (4.0–6.0)	− 1.5 to 0.5	0.2
Winter iFGF	43 (36–56)	41 (35–49)	−5 to 8	0.14
Summer iFGF	46 (40–60)	47 (38–52)	−6 to 6	0.3
Winter FGFc	95 (76–136)	85 (73–112)	− 12 to 38	0.08
Summer FGFc	93 (77–114)	90 (72–124)	− 15 to 18	0.3
Winter Klotho	682 (517–817)	677 (553–964)	− 182 to 134	0.6
Summer Klotho	588 (491–743)	732 (571–976)	− 257 to 16	0.08
Winter Ferritin	103 (58–214)	73 (24–170)	−34 to 75	0.2
Summer Ferritin	98 (44–185)	90 (35–148)	−32 to 67	0.5
Winter 125(OH)_2_D	148 (116–181)	139 (121–155)	−19 to 25	0.4
Summer 125(OH)_2_D	168 (133–201)^**+**^	176 (147–204)^**^	−27 to 27	0.7
Restricted to subjects who provided both a winter and summer specimen, For all analytes below *n* = 38 for RRMS and *n* = 23 for HC				
Winter 25OHD	59 (38–91)	47 (37–79)	−17 to 32	0.4
Summer 25OHD	87 (70–108)^**^	81 (70–92)^**^	−6 to 18	0.4
Winter PTH	4.5 (3.8–6.1)	5.8 (4.0–6.6)	−1.7 to 0.3	0.09
Summer PTH	4.7 (3.9–5.7)	5.0 (4.0–6.0)	−1.5 to 0.5	0.3
Winter iFGF	45 (36–59)	45 (35–50)	−6 to 9	0.3
Summer iFGF	46 (40–60)	49 (40–52)	−6 to 5	0.4
Winter FGFc	93 (77–134)	96 (76–123)	− 23 to 24	0.4
Summer FGFc	93 (77–114)	90 (75–134)	− 15 to 17	0.5
Winter Klotho	681 (523–749)	677 (569–1034)	− 154 to 104	0.5
Summer Klotho	588 (491–743)	725 (563–984)	− 231 to 27	0.1
Winter Ferritin	108 (60–224)	62 (21–153)	−4 to 87	0.06
Summer Ferritin	98 (44–188)	89 (32–134)	−25 to 67	0.4
Winter 125(OH)_2_D	150 (114–193)	148 (126–160)	−16 to 31	0.5
Summer 125(OH)_2_D	168 (133–201)^**++**^	177 (145–204)^*^	−27 to 27	0.7

Abbreviations: *IQR* interquartile range

*P*: ^*^ < 0.05, ^**^ < 0.005, ^***^ < 0.0005, ^**+**^ 0.07, ^**++**^ 0.23 for within-cohort, winter versus summer values for 25OHD and 1,25(OH)_2_D tabulated above

### PTH and iFGF23

Pairs analysis revealed that subjects with RRMS had lower plasma PTH than HC in winter and summer (Fig. 2, Table 2). For example, the median winter within-pair difference (RRMS-HC) in plasma PTH was − 1.6 pmol/L (*P* = 0.005). To put the magnitude of this difference in context, it is over half the magnitude of the HC IQR for winter plasma PTH (Table 1).

**Fig. 2:** Within-pair differences (RRMS-HC) in plasma PTH

**Table 2:** Pairs analyses (subject with RRMS minus HC friend)

Chemical	Median difference (IQR)	95% CI for median difference	*P* value
Analyses of all pairs: *n* = 28 pairs (winter) 21–23 (summer)			
Winter 25OHD	17 (−8 to 48)	−5 to 37	0.03
Summer 25OHD	11 (− 12 to 41)	−9 to 35	0.09
Winter PTH	− 1.6 (− 2.6 to 0.6)	−2.4 to 0.5	0.005
Summer PTH	−1.1 (−2.0 to 0.7)	−1.8 to 0.5	0.04
Winter iFGF	5 (−6 to 18)	−3 to 15	0.04
Summer iFGF	4 (−6 to 15)	−5 to 13	0.14
Winter FGFc	7 (−25 to 49)	−15 to 45	0.15
Summer FGFc	−4 (−34 to 29)	−26 to 19	0.7
Winter Klotho	−58 (− 314 to 147)	− 252 to 88	0.4
Summer Klotho	− 206 (− 469 to 117)	− 386 to 40	0.05
Winter Ferritin	50 (−58 to 89)	−45 to 63	0.3
Summer Ferritin	27 (−57 to 90)	−36 to 79	0.4
Winter 125(OH)_2_D	6 (−20 to 29)	−9 to 18	0.4
Summer 125(OH)_2_D	−4 (−50 to 18)	−42 to 15	0.5
BMI	−1.4 (−5.6 to 4.4)	−4.5 to 2.4	0.8
Restricted to pairs who provided winter and summer specimens: *n* = 21–23 pairs			
Winter 25OHD	7 (−8 to 51)	−6 to 46	0.08
Summer 25OHD	11 (−12 to 41)	−9 to 35	0.09
Winter PTH	−1.5 (−2.6 to 0.6)	−2.5 to 0.6	0.02
Summer PTH	−1.1 (−2.0 to 0.7)	− 1.8 to 0.5	0.04
Winter iFGF	6 (−4 to 16)	−3 to 15	0.05
Summer iFGF	4 (−6 to 15)	−5 to 13	0.14
Winter FGFc	3 (−36 to 47)	−25 to 42	0.4
Summer FGFc	−4 (−34 to 29)	−26 to 19	0.7
Winter Klotho	−81 (− 349 to 96)	− 297 to 88	0.2
Summer Klotho	−206 (−469 to 117)	−386 to 40	0.05
Winter Ferritin	52 (−54 to 164)	−21 to 87	0.13
Summer Ferritin	27 (−57 to 90)	−36 to 79	0.4
Winter 125(OH)_2_D	2 (−32 to 30)	−19 to 22	0.7
Summer 125(OH)_2_D	−4 (−50 to 18)	−42 to 15	0.5

No significant differences were detected across season

*Abbreviations*: *IQR* interquartile range

In subjects with RRMS, plasma iFGF23 was the same as or higher than in HC (Fig. 3, Table 2). For example, the median winter within-pair difference (RRMS-HC) in plasma iFGF23 was 5 pg/mL (*P* = 0.04). To put the magnitude of this difference in context, it approximates one third the magnitude of the HC IQR for winter plasma iFGF23 (Table 1).

**Fig. 3:** Within-pair differences (RRMS-HC) in plasma iFGF23

### Ratio of serum 1,25(OH)2D to 25OHD

As PTH increases and iFGF23 reduces the activity of renal 1-alpha hydroxylase, which synthesises serum 1,25(OH)_2_D from serum 25OHD, (and as PTH reduces and iFGF23 increases the activity of renal 24-hydroxylase which degrades serum 1,25(OH)_2_D) we compared the ratio of the serum concentrations of 1,25(OH)_2_D and 25OHD between RRMS and HC. Subjects with RRMS had a lower ratio of serum 1,25(OH)_2_D (pmol/L) to serum 25OHD (nmol/L). The median winter within-pair difference (RRMS-HC) in this ratio was − 0.7 (*P* = 0.013, 95% CI -1.2 to − 0.3, *n* = 28 pairs) (Fig. 4). To put the magnitude of this difference in context, it is over one third the magnitude of the HC IQR for the winter ratio of serum 1,25(OH)_2_D (pmol/L) to serum 25OHD (nmol/L); as the median (IQR) HC winter ratio was 3.1 (2.0–3.8).

**Fig. 4:** Within-pair differences (RRMS-HC) in the serum 1,25(OH)_2_D to 25OHD ratio

In the smaller sample of summer pairs, the median within-pair difference (RRMS-HC) of the ratio of serum 1,25(OH)_2_D to serum 25OHD was − 0.3, which did not reach significance (*P* = 0.07, 95% CI -0.9 to 0.1, *n* = 22 pairs) (Fig. 4), potentially because of the smaller sample size.

### Examination of potential confounders

The RRMS cohort contained a higher proportion of females, and plasma PTH may vary with renal function and plasma FGF23 with serum magnesium and ferritin (Takeda et al. 2011; Braithwaite et al. 2012; Durham et al. 2007). Therefore, we explored post-hoc whether the lower plasma PTH and paradoxically similar or higher plasma iFGF23 in subjects with RRMS could be due to confounding by sex or serum creatinine, magnesium, ferritin or 25OHD.

Either for all subjects combined, or within the separate RRMS and HC cohorts, plasma PTH and plasma iFGF23 did not differ by sex and in winter neither was associated with serum creatinine, which itself did not differ between RRMS and HC.

The median within-pair difference (RRMS-HC) in serum magnesium was not significantly different from zero (both in winter and summer). The median within-pair difference (RRMS-HC) in serum ferritin was not significantly different from zero (both in winter and summer). Furthermore, there was no correlation between within-pair differences in plasma iFGF23 and within-pair differences in serum ferritin.

The bivariate relationship between serum 25OHD and plasma PTH was weak (Fig. 5). Winter serum 25OHD correlated inversely with winter plasma PTH for all subjects combined (*r* = − 0.27, *P* = 0.02) and within the RRMS (*r* = − 0.32, *P* = 0.03) but not the HC cohort (*r* = − 0.06, *P* = 0.7). In summer, serum 25OHD did not correlate with plasma PTH. Furthermore, serum 25OHD did not correlate with plasma iFGF23, plasma FGF23c, plasma klotho or serum ferritin.

**Fig. 5:** Plasma PTH and Serum 25OHD Plasma PTH in winter (open circles) and summer (solid circles) plotted against serum 25OHD for subjects who provided both winter and summer venepuncture. Three outliers (serum 25OHD > 150 nM) were excluded to enlarge the scale of the X-axis

In summary, lower plasma PTH and similar or higher plasma iFGF23 in RRMS compared with HC subjects was not due to confounding by sex or serum creatinine, magnesium, ferritin or 25OHD.

## Discussion

We present evidence for dysequilibrium of the PTH-FGF23-vitamin D axis in RRMS. Subjects with RRMS had lower plasma PTH concentrations than HC, yet their plasma iFGF was the same as or higher than HC. In winter, when vitamin D nutrition was lowest, they had a lower serum 1,25(OH)_2_D to 25OHD ratio and in summer they failed to demonstrate a rise in serum 1,25(OH)_2_D, as observed in HC. These findings are consistent with our initial hypothesis that there is suppression of PTH in RRMS, associated with higher serum FGF23. The magnitude of this dysequilibrium was large. The median winter RRMS-HC difference in plasma PTH exceeded half the HC IQR for winter plasma PTH and the median winter RRMS-HC difference in plasma iFGF23 approximated a third of the HC IQR for winter iFGF23. Similarly, the median winter RRMS-HC difference in the ratio of serum 1,25(OH)_2_D to 25OHD exceeded a third of the HC IQR for the winter value of this ratio.

Dysequilibrium of the PTH-FGF23-vitamin D axis data exhibited internal consistency. Thus, lower plasma PTH and higher plasma iFGF23 observed in RRMS would be expected to lead to lower renal 1-alpha hydroxylase activity in RRMS and thus decreased synthesis of serum 1,25(OH)_2_D from 25OHD (Tanaka and DeLuca 1981; Bacchetta et al. 2013; Shimada et al. 2004; Shimada et al. 2005). Lower plasma PTH and higher plasma iFGF23 in RRMS would also be expected to lead to higher renal 24-hydroxylase activity in RRMS with increased degradation of serum 1,25(OH)_2_D (Tanaka and DeLuca 1981; Bacchetta et al. 2013; Shimada et al. 2004; Shimada et al. 2005). Accordingly, the winter serum 1,25(OH)_2_D to 25OHD ratio was lower in RRMS than HC and subjects with RRMS did not demonstrate the expected summer rise in serum 1,25(OH)_2_D observed in HC. Unlike the Finnish study of Soilu-Hänninen et al. (Soilu-Hänninen et al. 2008), we did not find a lower winter serum calcium concentration in RRMS, which might be explained by the fact that the winter serum 25OHD was higher in the Australian subjects. Irish researchers examined PTH at low levels of 25OHD (Lonergan et al. 2011; McKenna et al. 2018). In one study (Lonergan et al. 2011) a significant inverse correlation of PTH with 25OHD was present in controls but not in people with MS. Those studies, however, did not report plasma calcium and their MS cohort grouped primary progressive and secondary progressive MS together with RRMS (Lonergan et al. 2011; McKenna et al. 2018). Blau and Collins (Blau and Collins 2015) wrote “The action of FGF23 on the parathyroid gland has been reported to suppress PTH secretion in vitro and in rodent models, but demonstration of a similar effect in humans is lacking.” Although our findings are correlative they are consistent with a physiological effect of FGF23 to suppress the parathyroid glands in RRMS.

We were not able to determine if dysequilibrium of the PTH-FGF23-vitamin D axis precedes or follows the pathophysiology of RRMS. It is interesting, however, that while we find differences (RRMS vs HC) in the levels of hormones (PTH and iFGF23) that regulate the activity of the enzymes 1-alpha hydroxylase and 24-hydroxylase, which respectively synthesise and degrade the potent vitamin D metabolite 1,25(OH)_2_D, others find differences between people with MS versus HC in the genes coding for these same enzymes (Pierrot-Deseilligny and Souberbielle 2017). This certainly raises the possibility that dysequilibrium of the PTH-FG23-vitamin D axis could have a pathogenic role. In addition, because PTH and FGF23 also regulate extra-renal 1-alpha hydroxylase in innate and adaptive immune cells, (for example see Ref Bacchetta et al. 2013) this dysequilibrium has the potential to modify immune-inflammatory processes in MS via autocrine as well as endocrine vitamin D metabolism, in keeping with evidence that impaired vitamin D nutrition is associated with MS (Pierrot-Deseilligny and Souberbielle 2017; Munger et al. 2006; van der Mei et al. 2007; Simpson Jr et al. 2010).

It will be important to determine whether plasma PTH and plasma iFGF23 could be used as biomarkers to identify individuals at risk for RRMS or predict disease course and response to therapy. It will also be important to determine whether there is dysequilibrium in the PTH-FGF23-vitamin D axis in other autoimmune diseases such as type 1 diabetes, systemic lupus erythematosus and rheumatoid arthritis that exhibit an incidence or disease activity which correlates with vitamin D nutrition (Munger et al. 2013; Watad et al. 2017).

This study has several limitations. Not all of the differences between RRMS and HC demonstrated by within-pair analysis were seen in comparison of RRMS and HC cohort medians. Furthermore, not all subjects with RRMS recruited a HC friend to the study. While cohort analyses have the advantage of larger sample size, analysis of RRMS-HC pairs may be more sensitive as it controls for pre-analytical specimen handling measurement error (each RRMS-HC friend pair attended the same specimen collection centre at the same time), which may contribute up to 50% of total analyte measurement error (Plebani 2006). To reduce analytical laboratory error, winter and summer specimens from each RRMS-HC pair were analysed within the same ELISA plate. In addition, we deliberately recruited HC from friends of the people with RRMS to minimise bias from unmeasured lifestyle, social and demographic variables that could potentially mask disease-specific differences. A further potential limitation is that we did not measure markers of inflammation, which could confound the interpretation of serum ferritin concentrations, if people with RRMS had more inflammation than HC. Lower serum ferritin concentrations have been associated with higher serum concentrations of FGF23c and iFGF23 (Braithwaite et al. 2012; Durham et al. 2007), but this relationship appears to be assay specific (Durham et al. 2007). In particular, the Kainos iFGF23 assay used in this study was not affected by low concentrations of serum ferritin (Durham et al. 2007). Hence, potential confounding of serum ferritin by inflammation in the RRMS cohort would not explain higher RRMS plasma concentrations of iFGF23 in this study. Finally, the fact that some subjects chose not to return for summer venepuncture may have introduced bias into the study. However, subjects were recruited both from hospital MS clinics and from the community, supporting the generalizability of the results.

## Conclusions

This study revealed a dysequilibrium of the PTH-FGF23-vitamin D axis in RRMS, with lower plasma PTH, higher plasma iFGF23 and a lower serum 1,25(OH)_2_D to 25OHD ratio in RRMS compared with HC subjects. This dysequilibrium is consistent with the study hypothesis that in RRMS there is suppression of the parathyroid glands by inappropriately high plasma concentrations of iFGF23. The basis of this dysequilibrium may provide insight into the pathogenesis of RRMS and requires further investigation.

## Abbreviations

1,25(OH)_2_D: 1,25-dihydroxyvitamin D
25OHD: 25-hydroxyvitamin D
CI: Confidence interval
FGF23: Fibroblast growth factor 23
FGFc: c-terminal fibroblast growth factor 23
HC: Healthy control(s)
iFGF23: Intact fibroblast growth factor 23
IQR: Interquartile range
Klotho: Soluble alpha klotho
PTH: Parathyroid hormone
RRMS: Relapsing remitting multiple sclerosis
